# Personality traits that associate with sustainable behaviors perceived by individuals

**DOI:** 10.1002/brb3.3147

**Published:** 2023-07-11

**Authors:** Zhao Longlong

**Affiliations:** ^1^ School of Philosophy Renmin University of China Beijing China; ^2^ Department of Political Science University College London London UK

**Keywords:** HEXACO, personality traits, quantitive relationship, regression analysis, sustainable behaviors perceived by individuals

## Abstract

**Introduction:**

There is relatively little research on the association between personality traits and sustainable behaviors. So, this research was designed to differentiate associations between the six personality traits and sustainable behaviors perceived by individuals.

**Methods:**

A total of 1420 residents in a community of Nanjing participated in this survey. With the help of HEXACO‐60 and SBPI‐9, participants’ personality traits and the performance of sustainable behaviors perceived by individuals were measured. Subsequently, assisted by regression analysis, the quantitive relationship between HEXACO and sustainable behaviors perceived by individuals was explored.

**Results:**

Honesty–humility (H–H), extraversion (X), consciousness (C), and openness to experience (O) are positively associated with sustainable behaviors perceived by individuals, whereas emotionality (E) and agreeableness (A) are negatively associated with it.

**Conclusions:**

HEXACO have a significant association with sustainable behaviors perceived by individuals. Additionally, H–H, E, X, A, C, and O could explain 44.2% of changes in sustainable behaviors perceived by individuals.

## 1 INTRODUCTION

Personality traits have a certain association with people's attitudes and behavior habits (Nyhus & Pons, 2005). There are obvious differences in attitudes and behavior habits between two people with different personalities (Thielmann et al., 2020). Conversely, behavioral manners might shape or strengthen a person's personality traits to a certain extent (Thielmann et al., 2020). The relationship between personality traits and personal behavior is an important research topic in the field of psychology, and it has attracted the attention of many researchers (Zhao, 2022). In specific scenarios, exploring the association between the two might expand the current research content and provide some references for the solution of some practical problems (Dilchert & Ones, 2008).

Green development has become an essential topic that scholars in recent years have hotly debated (Wang & Jiang, 2020). Different from the traditional development manner, green development is a new model, which is committed to building a harmonious coexistence between human beings and nature, emphasizing promoting economic growth and social development through energy conservation, emission reduction, and environmental protection (Soutter & Boag, 2019; Soutter et al., 2020; Thielmann et al., 2020; Wang & Jiang, 2020).

As an integral approach to achieving green development, promoting sustainable behaviors attracts growing research attention (Biswas et al., 2022). Sustainable behaviors is a collective term for a series of pro‐environmental actions, with “low energy consumption, low pollution, and low emissions” being its main goals and principles (Foster et al., 2022; Nezlek, 2022; Soutter & Boag, 2019; Soutter et al., 2020; Sovacool et al., 2022). The common sustainable behaviors are recycling personal idle items timely (Johnstone & Lindh, 2022), sorting waste when disposed of (Zhao et al., 2022), preparing eco‐friendly shopping bags in advance before shopping (Luo et al., 2022), and actively participating in various low‐carbon environmental protection–related activities (Biswas et al., 2022).

Research studies around the psychological factors that associate with individual behaviors concentrate on five aspects, namely, values (Ali et al., 2022), attitude (Mckenzie‐Mohr, 2000), self‐efficacy (Foster et al., 2022), cognition (Sovacool et al., 2022), preferences (Smith et al., 2022), and personality traits (Ali et al., 2022). However, the association between personality traits and sustainable behaviors has not been given enough attention (Foster et al., 2022). In particular, there are few studies on investigating the relationship between sustainable behavior and personality traits in the scenario of China (mainland).

To control the intensification of environmental pollution and promote green development, many cities in China have successively issued a series of policies related to sustainable development (Wu et al., 2020). Nanjing, the capital of Jiangsu Province, began exploring new paths to low‐carbon development in 2016 (Zhang, Luo, et al., 2022; Zhang, Xie, et al., 2022). After more than 4 years of effort, Nanjing has achieved relatively remarkable results in green development. Currently, the Nanjing Municipal Government is actively advocating for more citizens and social organizations to participate in activities to control greenhouse gases and reduce carbon emissions, using business incentives, policy incentives, and trading mechanisms (Yang & Wei, 2020). Thus, investigating personality traits of citizens in Nanjing that associate with sustainable behaviors perceived by individuals is an adequate choice that matches the current trend.

Therefore, this paper takes more than 1000 residents from community A in Nanjing, Jiangsu Province, as the primary research subject, and with the help of HEXACO‐60 and SBPI‐9, residents’ personality traits and sustainable behaviors perceived by themselves were explored. Then, the quantitative relationship between the two was differentiated and studied in detail. In this way, it is possible to distinguish what personality traits are associated with better performance of pro‐environmental actions in the scenario of China. Thus, specific suggestions can be provided for promoting sustainable behaviors from the perspective of personality characteristics.

## 2 MAIN HYPOTHESIS

The prosocial behavior is an act that meets the social expectations currently and positively impacts other people or societies (Kirakozian, 2017; Xu et al., 2018). Most scholars tend to divide prosocial behaviors into three types roughly (Andersson & Stage, 2018). The first category is altruistic behavior, which is the kind of voluntary behavior that is beneficial to others but has no apparent benefit to the actors and even causes losses to the actors (Sundqvist‐Andberg & Åkerman, 2021). The second category is helping behavior, which is intended to help another person or a group with or without reward (Minelgaitė & Liobikienė, 2019). The third category is reciprocal behavior, often seen as a behavioral equivalent exchange between individuals, which is, in most cases, positive and will bring some equivalent benefit to both (Sundqvist‐Andberg & Åkerman, 2021). Meanwhile, a behavioral equivalent exchange can also be unfavorable, causing some equivalent losses to both (Minelgaitė & Liobikienė, 2019). The sustainable behavior refers to a series of individual behaviors directed by “low energy consumption, low pollution, and low emissions” (Sabbir & Taufique, 2022), and it has a high consistency with altruistic behavior (Smith et al., 2022). This study chose to investigate the sustainable behaviors perceived by individuals (last 2 weeks) of urban residents after the green development policy had been implemented for 7 years, which is a rational decision after considering the variability and relative stability of the sustainable behavior (Bertoldi, 2020).

Recently, some researchers conducted a series of exploratory studies around HEXACO (Wertag & Bratko, 2018). In 2010, Ashton and Lee (2010) further divided the six personality traits in HEXACO into two categories when exploring the relationship between HEXACO and prosocial behavior. The first category mainly contains three personality traits: H–H, E, and A (Thielmann et al., 2020). Meanwhile, X, C, and O fall into the second category (Van Witteloostuijn et al., 2017; Wertag & Bratko, 2018). They found that H–H, E, and A could make outstanding contributions to predicting prosocial behavior (Ashton & Lee, 2010). However, X, C, and O do not seem to have a significant relationship with altruistic motives or behavior (Ashton & Lee, 2010).

Subsequently, Hilbig et al. (2014) conducted another study on the relationship between personality traits and prosocial behavior. From their research results, H–H, E, and A are strong predictors of prosocial behavior, whereas X, C, and O are proven to have a specific impact on prosocial behavior (Hilbig et al., 2014). This conclusion was also verified by Wertag and Bratko (2016). Through research, Wertag and Bratko (2019) found that H–H, E, X, A, C, and O all significantly influence prosocial behavior. However, from the degree of influence on prosocial behavior and the strength of explanation, Dark Triad (mainly including Machiavellianism, subclinical narcissism, and psychopathy) is better than HEXACO (Wertag & Bratko, 2019). And then Van Witteloostuijn et al. (2017) argued that there was a significant correlation between H–H/E/A/C/O and prosocial motive. After analyzing the relationship between personality traits and prosocial behavior in the scenario of economic games, Thielmann et al. (2020) found that H–H was the most robust predictor of prosocial behavior in the dictator game, trust game, prisoner's dile game, and commons dilemma. However, in the ultimatum game, A took the place of the most robust predictor (Thielmann et al., 2020).

Next, they argued that personality traits could be accountable factors for prosocial behavior (Thielmann et al., 2020). In short, it is more likely that there is a significant correlation between H–H/E/A and prosocial behavior. In contrast, the possibility of a significant association between C and prosocial behavior is relatively limited. As for X and O, from the current research results, it can only be inferred that there may be a limited association between X/O and altruistic behavior, but the significance of this association is complex.

Meanwhile, with the help of meta‐analysis, Soutter et al. (2020) directly pointed out a significant correlation between H–H/A/C and pro‐environmental behaviors. Subsequently, Nezlek and Cypryańska (2023) further proposed a significant positive correlation between openness to experience/neuroticism/agreeableness/extroversion/conscientious and certain self‐reported climate change mitigation behaviors. Thus, considering the distinctions and connections between the Big Five and HEXACO, as well as the relationship between personality traits and altruistic/prosocial behaviors described above, it is likely to predict that H–H/E/X/A/C/O is associated with sustainable behaviors perceived by individuals significantly.

Hypothesis 1 H–H/E/X/A/C/O associates with sustainable behaviors perceived by individuals significantly.

## 3 DATA AND METHODOLOGY

### 3.1 Participants

One thousand four hundred and twenty questionnaires were distributed, but only 1255 were recycled (the recovery rate is 88.38%). Of the recycled questionnaires, 35 copies were not accomplished by the participants. In other words, the 35 questionnaires had 2 or 3 questions not answered by their corresponding fillers. Therefore, these five questionnaires were judged to be invalid. The fillers of the 1220 valid questionnaires were all Chinese or, more precisely, Chinese residents of community A in Nanjing, Jiangsu Province (located in the south of China). All participants were randomly selected by the authors in community A using the convenience sampling method. After filling out the questionnaire, each filler received a souvenir provided by the author.

### 3.2 Materials

In order to protect the privacy of the questionnaire fillers, none of the questionnaires collected information that could identify the participants. There are two paper questionnaires used in this survey. The first questionnaire consisted of two parts. The first part of the questionnaire focused on investigating participants’ gender (with “1” representing male and “2” representing female), age (with “1” representing 25–35‐year old, “2” representing 36–46‐year old, “3” representing 47–57‐year old, “4” representing 58–68‐year old, and “5” representing over 68‐year old), an education level (with “1” standing for below high school degree, “2” standing for a high school degree, “3” standing for the bachelor's degree, “4” standing for the master's degree, and “5” standing for the PhD), and annual income (with “1” standing for less than 12,000 pounds, “2” standing for 12,001–24,000 pounds, “3” standing for 24,001–36,000 pounds, “4” standing for 36,001–48,000 pounds, and “5” standing for over 48,001 pounds).

The second part of the first questionnaire was SBPI‐9, created by the Nanjing Municipal Government in the Low Carbon Living Initiative (Bi et al., 2011; Zhang, Luo, et al., 2022; Zhang, Xie, et al., 2022). It divides sustainable behaviors into nine facets, namely, the choice of public transportation, the recycling of idle items, the saving of water/electricity/natural gas, the separation of individual/household waste, the purchase of energy‐saving household appliances, the preparation of environmentally friendly shopping bags, the selection of clothing fabrics, the purchase of electronic products, and the participation in environmental protection activities. (See Appendix 1 for the performance of residents’ sustainable behaviors.) Each question is a multiple‐choice question using the Likert type of scale, and the corresponding value increases from 1 (representing “strongly disagree”) to 5 (representing “strongly agree”).

The second questionnaire was the HEXACO‐60 Inventory created by Lee and Ashton (2018). Because HEXACO‐60 has a Chinese version, the authors directly used the Chinese version of HEXACO‐60 in this survey after obtaining the creators’ consent. There are 60 questions in this part, and every 10 questions correspond to a personality trait in HEXACO (See Appendix 1 for the correspondence between personality traits and topics.), such as H–H is measured by the 6th, 30th, 54th, 12th, 36th, 60th, 18th, 42nd, 24th, and 48th question. Meanwhile, X is measured by the 4th, 28th, 52nd, 10th, 34th, 58th, 16th, 40th, 22nd, and 46th question. Each question is a multiple‐choice question using the Likert Type of Scale, and the corresponding value increases from 1 (representing “strongly disagree”) to 5 (representing “strongly agree”).

### 3.3 Procedure

At the east gate of community A, the first questionnaire was distributed. The author handed out each resident who completed the questionnaire a numbered postcard. The number on each postcard matches the code of the questionnaire filled out by every participant. They were then told to come to the east gate of community A 2 weeks later with the numbered postcard to complete a second questionnaire. After completing the second questionnaire (HEXACO‐60), they received a souvenir provided by the author. Each participant was given a numbered postcard to accurately link together two questionnaires filled out by the same participant.

After that, the authors tested Cronbach's *α* of honesty–humility, emotionality, extraversion, agreeableness, consciousness, openness to experience, and the performance of residents’ sustainable behaviors, with the help of Stata, a software that can be used for data analysis, and found that they were .87, .83, .81, .85, .82, .86, and .84, respectively. It can be seen that the questionnaire on personality traits and the performance of residents’ sustainable behaviors has a high degree of consistency.

### 3.4 Findings

According to the statistics, 1255 Nanjing citizens participated in the survey, of which 1220 questionnaires were identified as valid. The basic information of all valid questionnaires could be introduced from the following aspects. First, 670 men (54.92%) and 550 women (45.08%) participated in the survey. Second, 196 participants (20.08%) are 25–35‐year old (including 25 and 35), 255 participants (20.90%) are aged 36–46‐year old (including 36 and 46), 312 participants (25.61%) are 47–57‐year old (including 47 and 57), 270 participants are (22.13%) 58–68‐year old (including 58 and 68), 138 participants (11.27%) are over 68‐year old. Third, most of the respondent's education level was concentrated in high school degree, with about 345 individuals (28.28%), followed by the master's degree, with about 22.34% individuals; the bachelor's degree, with about 18.85% individuals; and the below high school degree, with about 18.24% individuals; the PhD degree, with about 12.30% individuals. Fourth, the annual income (before tax) of residents participating in the survey was mainly concentrated at less than 12,000 pounds (27.87%), followed by 12,001–24,000 pounds (23.36%), 24,001–36,000 pounds (19.67%), 36,001–48,000 pounds (17.42%), and over 48,001 pounds (11.68%). Additionally, Table 1 presents a statistical description of the main variables.

**TABLE 1:** Statistical description of main variables.

Variable	Mean	Standard deviation	Minimum	Maximum
Sustainable behaviors	3.312	1.130	1	5
Openness to experience	2.911	.809	1	4.1
Emotionality	2.847	1.115	1	5
Agreeableness	2.808	.962	1	4.3
Honesty–humility	3.545	.728	2.1	5
eXtraversion	3.088	1.269	1	4.8
Consciousness	2.868	.917	1	4.5
Sustainable behavior‐01	3.272	1.094	1	5
Sustainable behavior‐02	3.351	1.195	1	5
Sustainable behavior‐03	3.333	1.209	1	5
Sustainable behavior‐04	3.312	1.163	1	5
Sustainable behavior‐05	3.311	1.146	1	5
Sustainable behavior‐06	3.312	1.129	1	5
Sustainable behavior‐07	3.332	1.159	1	5
Sustainable behavior‐08	3.252	1.108	1	5
Sustainable behavior‐09	3.333	1.184	1	5

*Note*: Sustainable behavior‐01, sustainable behavior‐02, sustainable behavior‐03, sustainable behavior‐04, sustainable behavior‐05, sustainable behavior‐06, sustainable behavior‐07, sustainable behavior‐08, and sustainable behavior‐09 represented the 1st–9th question in the SBPI‐9 Inventory. Additionally, there were nine aspects of sustainable behaviors. Then, the value of sustainable behaviors = (sustainable behavior‐01 + sustainable behavior‐02 + sustainable behavior‐03 + sustainable behavior‐04 + sustainable behavior‐05 + sustainable behavior‐06 + sustainable behavior‐07 + sustainable behavior‐08 + sustainable behavior‐09)/9.

With the help of a partial correlation analysis, this paper tests the association between HEXACO and sustainable behaviors perceived by individuals (including its nine facets), and the results are shown in Table 2 (from sections one to ten). Based on the results presented in Table 2, it can be inferred that H–H/E/A/C/O has a positive association with sustainable behaviors perceived by individuals (the nine facets are included) significantly. In comparison, there is a nonsignificant association between X and sustainable behaviors perceived by individuals (containing its nine facets).

**TABLE 2:** The results of a partial correlation analysis.

Section one							
Variables	Sustainable behaviors	Openness to experience	Emotionality	eXtraversion	Agreeableness	Honesty–humility	Consciousness
Sustainable behaviors	1.000						
Openness to experience	.373***	1.000					
Emotionality	.299***	.358***	1.000				
eXtraversion	.015	−.063**	−.318***	1.000			
Agreeableness	.289***	.140***	.356***	.022	1.000		
Honesty–humility	.506***	.132***	.584***	−.322***	.519***	1.000	
Consciousness	.356***	.087***	.043	−.057**	.132***	.221***	1.000

Section two							
Variables	Sustainable behavior‐01	Openness to experience	Emotionality	eXtraversion	Agreeableness	Honesty–humility	Consciousness
Sustainable behavior‐01	1.000						
Openness to experience	.366***	1.000					
Emotionality	.291***	.358***	1.000				
eXtraversion	.023	−.063**	−.318***	1.000			
Agreeableness	.300***	.140***	.356***	.023	1.000		
Honesty–humility	.500***	.132***	.584***	−.322***	.519***	1.000	
Consciousness	.299***	.087***	.043	−.057**	.132***	.221***	1.000

Section three							
Variables	Sustainable behavior‐02	Openness to experience	Emotionality	eXtraversion	Agreeableness	Honesty–humility	Consciousness
Sustainable behavior‐01	1.000						
Openness toexperience	.376***	1.000					
Emotionality	.308***	.358***	1.000				
eXtraversion	.005	−.063**	−.318***	1.000			
Agreeableness	.256***	.140***	.356***	.023	1.000		
Honesty–humility	.481***	.132***	.584***	−.322***	.519***	1.000	
Consciousness	.357***	.087***	.043	−.057**	.132***	.221***	1.000

Section four							
Variables	Sustainable behavior‐03	Openness to experience	Emotionality	eXtraversion	Agreeableness	Honesty–humility	Consciousness
Sustainable behavior‐03	1.000						
Openness to experience	.365***	1.000					
Emotionality	.288***	.358***	1.000				
eXtraversion	.006	−.063**	−.318***	1.000			
Agreeableness	.271***	.140***	.356***	.023	1.000		
Honesty–Humility	.494***	.132***	.584***	−.322***	.519***	1.000	
Consciousness	.369***	.087***	.043	−.057**	.132***	.221***	1.000

Section five							
Variables	Sustainable behavior‐04	Openness to experience	Emotionality	eXtraversion	Agreeableness	Honesty–humility	Consciousness
Sustainable behavior‐04	1.000						
Openness to experience	.340***	1.000					
Emotionality	.288***	.358***	1.000				
eXtraversion	.016	−.063**	−.318***	1.000			
Agreeableness	.313***	.140***	.356***	.023	1.000		
Honesty–humility	.522***	.132***	.584***	−.322***	.519***	1.000	
Consciousness	.400***	.087***	.043	−.057**	.132***	.221***	1.000

Section six							
Variables	Sustainable behavior‐05	Openness to experience	Emotionality	eXtraversion	Agreeableness	Honesty–humility	Consciousness
Sustainable behavior‐05	1.000						
Openness to experience	.372***	1.000					
Emotionality	.265***	.358***	1.000				
eXtraversion	.025	−.063**	−.318***	1.000			
Agreeableness	.221***	.140***	.356***	.023	1.000		
Honesty–humility	.445***	.132***	.584***	−.322***	.519***	1.000	
Consciousness	.311***	.087***	.043	−.057**	.132***	.221***	1.000

Section seven							
Variables	Sustainable behavior‐06	Openness to experience	Emotionality	eXtraversion	Agreeableness	Honesty–humility	Consciousness
Sustainable behavior‐06	1.000						
Openness to experience	.387***	1.000					
Emotionality	.309***	.358***	1.000				
eXtraversion	.018	−.063**	−.318***	1.000			
Agreeableness	.271***	.140***	.356***	.023	1.000		
Honesty–humility	.487***	.132***	.584***	−.322***	.519***	1.000	
Consciousness	.302***	.087***	.043	−.057**	.132***	.221***	1.000

Section eight							
Variables	Sustainable behavior‐07	Openness to experience	Emotionality	eXtraversion	Agreeableness	Honesty–humility	Consciousness
Sustainable behavior‐07	1.000						
Openness to experience	.370***	1.000					
Emotionality	.314***	.358***	1.000				
eXtraversion	.007	−.063**	−.318***	1.000			
Agreeableness	.328***	.140***	.356***	.023	1.000		
Honesty–humility	.513***	.132***	.584***	−.322***	.519***	1.000	
Consciousness	.363***	.087***	.043	−.057**	.132***	.221***	1.000

Section nine							
Variables	Sustainable behavior‐08	Openness to experience	Emotionality	eXtraversion	Agreeableness	Honesty–humility	Consciousness
Sustainable behavior‐08	1.000						
Openness to experience	.345***	1.000					
Emotionality	.272***	.358***	1.000				
eXtraversion	.028	−.063**	−.318***	1.000			
Agreeableness	.288***	.140***	.356***	.023	1.000		
Honesty–humility	.507***	.132***	.584***	−.322***	.519***	1.000	
Consciousness	.345***	.087***	.043	−.057**	.132***	.221***	1.000

Section ten							
Variables	Sustainable behavior‐09	Openness to experience	Emotionality	eXtraversion	Agreeableness	Honesty–humility	Consciousness
Sustainable behavior‐09	1.000						
Openness to experience	.367***	1.000					
Emotionality	.299***	.358***	1.000				
eXtraversion	.005	−.063**	−.318***	1.000			
Agreeableness	.299***	.140***	.356***	.023	1.000		
Honesty–humility	.506***	.132***	.584***	−.322***	.519***	1.000	
Consciousness	.381***	.087***	.043	−.057**	.132***	.221***	1.000

*Note*: Sustainable behavior‐01 represented the first question in SBPI‐9 Inventory. Sustainable behavior‐02 represented the second question in SBPI‐9 Inventory. Sustainable behavior‐03 represented the third question in SBPI‐9 Inventory. Sustainable behavior‐04 represented the fourth question in SBPI‐9 Inventory. Sustainable behavior‐05 represented the fifth question in SBPI‐9 Inventory. Sustainable behavior‐06 represented the sixth question in SBPI‐9 Inventory. Sustainable behavior‐07 represented the seventh question in SBPI‐9 Inventory. Sustainable behavior‐08 represented the eighth question in SBPI‐9 Inventory. Sustainable behavior‐09 represented the ninth question in SBPI‐9 Inventory.

** Indicates that the correlation coefficient passes the significance test of the .05 level.

*** Indicates that the correlation coefficient passes the significance test of the .01 level.

This paper employs multiple linear regression analysis to clarify further the quantitative relationship between HEXACO and sustainable behaviors perceived by individuals. So, Model 1 was built. In Model 1, H–H, E, X, A, C, and O were treated as independent variables, and sustainable behaviors perceived by individuals were regarded as the dependent variable. According to the results presented in Table 3, H–H, X, C, and O positively impact sustainable behaviors perceived by individuals, whereas E and A negatively influence sustainable behaviors perceived by individuals robustly. That is to say that Hypothesis 1 could pass the test and be accepted.

**TABLE 3:** Regression results of Model 1.

	Coefficient	Standard error	*p*‐Value	*t*‐Value
Openness to experience	.451	.032	0.000	13.92
Emotionality	−.058	.029	.048	−1.98
eXtraversion	.181	.021	0.000	8.60
Agreeableness	−.583	.031	.056	−1.91
Honesty–humility	.834	.048	0.000	17.41
Consciousness	.283	.027	0.000	10.34
Constant	−1.997	.181	0.000	−11.00
Adjust *R*‐squared	.442			
Number of observations	1220			

Second, it can be figured out that in HEXACO, H–H is the strongest predictor for sustainable behaviors perceived by individuals, followed by A and O. In contrast, E is the weakest predictor. It means that the more prominent a person is in H–H/O in the sample surveyed, the better they are likely to perform in sustainable behaviors. Furthermore, the more significant a person's A/E is, the worse they are likely to perform in sustainable behaviors.

Next, in Model 1, H–H, E, X, A, C, and O provide a 44.2% explanation for the variance of sustainable behaviors perceived by individuals. Therefore, HEXACO can be used to predict and estimate an individual's performance of sustainable behaviors.

Moreover, in model 1, the “constant” value is negative. It may indicate that there might be some nonlinear connections between the independent variables and the dependent variable or the complex relationship between other independent variables and the dependent variable may generate it. In summary, the negative value of “constant” could not cause some obvious biases, as the values of the independent and dependent variables are from 1 to 5 (0 is not included).

## 4 DISCUSSION

This study found a significant association between the six personality traits included in HEXACO and sustainable behaviors perceived by individuals. This finding is consistent with previous findings (Alistair et al., 2020; Soutter et al., 2020; Thielmann et al., 2020). In particular, H–H and O are strong predictors of sustainable behaviors individuals perceive among the six personality traits, as Alistair et al. (2020) concluded. However, the negative association between E/A and sustainable behaviors perceived by individuals proved by this study is somewhat different from the previous findings of Nezlek and Cypryańska (2023).

During studying the relationship between personality and self‐reported climate change mitigation behaviors, with the help of the Big Five Inventory, Nezlek and Cypryańska (2023) found that neuroticism/agreeableness was positively associated with some climate change mitigation behaviors in the scenario of US collegians. However, there are some apparent differences between this paper and the above research in terms of the research object and the selected personality scale, so, understandably, the two have a bias in the conclusions.

In addition, according to the results of a partial correlation analysis, E/A was positively correlated with sustainable behaviors (including its nine facets). Nevertheless, according to the results presented by the regression analysis, the association between them became negative. The main reason for this change may be that the relationship between E/A and sustainable behaviors has been varied due to the influence of the traits in HEXACO other than E and A or the impact of the Chinese (mainland) cultural environment.

## 5 CONCLUSIONS

With the help of regression analysis, the association between personality traits and sustainable behaviors in Nanjing is studied. According to the analytic results, there is a positive association between H–H/X/C/O and sustainable behaviors perceived by individuals. Meanwhile, there is a negative association between E/A and sustainable behaviors perceived by individuals. Based on these, it can be inferred that when H–H/X/C/O shows a growth trend, sustainable behaviors perceived by individuals show a co‐increasing momentum, whereas when E/A presents a climb current, sustainable behaviors perceived by individuals present an adverse momentum.

In addition, it is worth mentioning that this paper is the first to conduct an empirical study of the association between personality traits and sustainable behaviors perceived by individuals in China (mainland). This paper not only distinguishes the quantitative relationship between the six personality traits and sustainable behaviors but also finds a new conclusion that for residents of community A in Nanjing, the more prominent their personality traits are in the perspective of E and A, the worse they are likely to perform in sustainable behaviors. Therefore, to improve the performance of individual sustainable behaviors in the scenario of China, it may be a benign option to weaken individuals’ traits called E and A. In addition, in the process of promoting and advocating sustainable behaviors, people with more obvious E and A characteristics are the ones who should be focused on, as they may perform worse.

There are two main limitations in this paper. To begin with, the performance of residents’ sustainable behaviors in the last 2 weeks is one of the focuses of this study. Although a resident's sustainable behaviors are relatively stable in the short term, it is not easy to accurately describe the general situation of the sustainable behavior in a given period by investigating the general status of their sustainable behaviors. It is difficult to operate an investigation that surveys residents’ sustainable behaviors multiple times in a given time; it makes sense to conduct such follow‐up surveys if possible. Second, the main subjects of this study (refers to the residents in communities) were randomly selected, and when the reality or situation is more complicated, there are certain shortcomings in the representativeness of the randomly selected samples.

Based on these, future research may develop in the following areas. First, collecting more panel data related to residents’ personality traits and sustainable behaviors, studying the changes in residents’ personality traits and sustainable behaviors over a specific period, and exploring whether there is a correlation between the two. Second, in the investigation process, gradually integrating more external factors, such as the impact of related incentive policies and management measures on residents’ personality traits and sustainable behaviors. Third, the specific process of how the residents’ personality traits impact their sustainable behaviors is needed to be explored further.

## CONFLICT OF INTEREST STATEMENT

The author has no conflict of interest.

## FUNDING INFORMATION

This paper is not supported by any funds.

### PEER REVIEW

The peer review history for this paper is available at https://publons.com/publon/10.1002/brb3.3147.

## Supporting information

Appendix 1

## Data Availability

Some or all data used during the study were provided by a research group led by the author. Anyone who wants to get access to the related datasets could send an email to jarryqotter@163.com.
